# Systematic Analysis of Tumor Microenvironment Patterns and Oxidative Stress Characteristics of Endometrial Carcinoma Mediated by 5-Methylcytosine Regulators

This article has been retracted.

**DOI:** 10.1155/2022/6431164

**Published:** 2022-09-21

**Authors:** Chunli Dong, Ling Dang, Xiaocui Gao, Renyan Xu, Hui Zhang, Xin Zhang

**Affiliations:** ^1^Department of Anesthesiology and Operation, The Second Affiliated Hospital of Xi'an Jiaotong University, China; ^2^Department of Obstetrics and Gynecology, The Second Affiliated Hospital of Xi'an Jiaotong University, China

## Abstract

As a widely distributed RNA methylation modification, m5C is involved in the regulation of tumorigenesis. Nevertheless, its fundamental process is not clear. This research sought to examine the genetic properties of the 5-methylcytosine (m5C) regulator in endometrial carcinoma, as well as the prognostic significance and impact of m5C regulators on oxidative stress. Therefore, the TCGA-UCEC data set was used to explore the characteristics of 17 RNAm5C-related genes in the transcriptome, genome, and regulatory network. The subtypes of RNAm5C in UCEC were identified based on the expression levels of 17 RNAm5C-related genes. The prognosis of RNAm5C-2 was significantly better than that of RNAm5C-1. Then, we examined the differences (variations) across various subtypes in terms of immune cell infiltration (ICI) as well as the expression of immune-related signal markers. The findings demonstrated that there were distinct variations in the infiltration level of immune cells in each subtype, which may be the reason for the differences in the prognosis of each subtype. In addition, the differentially expressed genes (DEGs) among RNAm5C subtypes of different UCEC tumors were identified, and the DEGs significant for survival were screened. After obtaining 34 prognostic genes, the dimensionality was reduced to construct an RNA methylation score (RS). As per the findings, RS is a more accurate marker for determining the prognosis for patients with endometrial cancer. The RS was used to categorize UCEC tumor samples, and these results led to the formation of high-score and low-score groups. The patients in the group with a high-RNA methylation score exhibited a survival time that was considerably longer in contrast with those in the group with a low-RNA methylation score. The capacity of RS to predict whether or not immunotherapy would be beneficial was explored further. In the group with a high-RNA methylation score, the objective response rate to the anti-PD-L1 therapy was substantially greater compared to that observed in the subgroup with a low-RNA methylation score. Additionally, there were variations across various RS groups in terms of clinical features, tumor mutation burden, and the infiltration level of immune cells. After binary tree analysis and PCR verification of 34 prognostic genes, it is finally found that the six genes of MAGOH3P, TRBJ2_3, YTHDF1P1, RP11_323D18.5, RP11_405M12.2, and ADAM30 are significantly overexpressed in cancer tissues. These genes can be used as potential biomarkers of endometrial cancer and provide data support for precise immunotherapy in UCEC tumors.

## 1. Introduction

Uterine corpus endometrial carcinoma (UCEC) is a prevalent cancer of the female reproductive system and has been ranked sixth among the most commonly diagnosed cancers in women, and the incidence rate is rising [1]. Patients diagnosed with early UCEC who have surgery have a five-year survival rate of between 74% and 91% [2, 3]. However, patients who have metastatic or recurrent endometrial cancer have a 5-year survival rate of just 20–26%, despite receiving radiotherapy and chemotherapeutic treatments [3, 4]. Therefore, endometrial cancer patients urgently need new and more effective treatment, and immune checkpoint inhibitors seem to offer new hope for UCEC therapy. In recent years, immunotherapy has become an effective treatment strategy for several solid cancers [5]. However, in UCEC, its efficacy is not satisfactory, which may be related to the microenvironment of UCEC itself. Therefore, it is imperative to examine the specific molecular and microenvironmental properties of UCEC to provide the groundwork for a therapy that could be successful. Although clinical characteristics and molecular biomarkers of UCEC patients have been utilized to make predictions about their clinical outcomes (prognosis), these strategies suffer from drawbacks. As a result, it is crucial to develop a unique predictive risk model to discover new prognostic indicators of UCEC and to anticipate the prognosis among patients who have UCEC.

The methylation modification of the fifth N of cytosine results in the formation of 5-methylcytidine also abbreviated as m5C. M5C methylation may be observed in a wide range of RNAs, which include tRNAs [6], mRNAs [7], sRNAs, and rRNAs [8]. Earlier research has demonstrated that m5C assumes a crucial regulatory function in a variety of mechanisms of gene expression, such as RNA output as well as ribosomal assembly and translation [9, 10]. Common m5C methylases include DNMT2 [11] and Nsun2 [12] and other related genes that have been identified but whose functions are not very clear. A growing body of research has concluded that m5C also performs an integral function in tumors. For example, YBX1 and NSUN2 target the m5C methylation site in the untranslated region of HDGF3 to promote the onset and progression of human bladder urothelial carcinoma, which may be linked to the mechanism that m5C can modulate cell division [13] and protein synthesis [14]. Nonetheless, very little is understood about the function of the m5C modulator in UCEC. As a result, it is imperative that the function of m5C in UCEC be analyzed thoroughly to offer a foundation for clinical application.

The tumor immune microenvironment usually assumes an integral function in cancer onset and progression [15, 16]. The heterogeneity of the immune microenvironment can affect many factors, such as patients' response to treatment and clinical outcomes [17, 18]. Immune cell infiltration has been demonstrated in previous research to have the capacity to control the advancement and metastasis of cancer in patients [19, 20]. However, the immune microenvironment in tumors is regulated by many factors. The significance of m5C as a factor in the microenvironment of tumors has been shown by an increasing number of studies. For example, the prognostic model established by m5C-related lncRNAs may predict the prognosis of lung adenocarcinoma and may be achieved by regulating the immune microenvironment [21], but the role of m5C-related genes in UCEC is not very clear, and whether to regulate its immune microenvironment needs further study. The relationship between the post-transcriptional modification of m5C-related mRNA and the tumor immune microenvironment in UCEC is unclear, and whether it affects the prognosis by reshaping the immune microenvironment is also unclear. At present, m5C has been linked to both the prognosis of patients with tumors and the immune microenvironment in a few different studies. Nevertheless, the main attention in these research studies is paid to a limited number of genes identified in the m5C maps of certain normal and cancer cells. There is currently a lack of information on certain gene properties and the prognostic significance of m5C-related genes in cancer, particularly UCEC.

To find a solution to this issue, this research employed the TCGA-UCEC data set to examine the properties of 17 genes associated with RNAm5C in the context of the genomic, transcriptomic, and regulatory network, and then we used the expression profile of 17 RNAm5C-related genes to identify RNAm5C subtypes. These subtypes have significant differences in the future, and the prognosis of RNAm5C-2 is significantly better than that of RNAm5C-1. After that, we examined the variations in the expression of immune cell infiltration (ICI) and immune-related signal markers that exist across the various RNAm5C subtypes. The findings demonstrated that there were considerable variations in terms of immune cell infiltration across these subgroups, which might also help to explain why there were remarkable differences in prognosis across the various subtypes. Additionally, the DEGs across distinct RNAm5C subtypes were identified, and the prognostic value of these genes was evaluated. 34 genes with prognostic significance were obtained. Based on this, an RNA methylation score (RS) was constructed. RS classified UCEC tumor samples into low- and high-score groups. Patients in the group with a high-RNA methylation score had a survival rate that was remarkably higher as opposed to that of patients in the group with a low-RNA methylation score. Furthermore, when compared to the low-RNA methylation score subgroup, the objective response rate to anti-PD-L1 therapy in the high-RNA methylation score group was substantially greater. We examined the variations in clinical features, tumor mutational burden, and the infiltration levels of immune cells that existed across all RS groups of UCEC tumors. After binary tree analysis and PCR verification of 34 prognostic genes, it was finally found that the six genes of MAGOH3P, TRBJ2_3, YTHDF1P1, RP11_323D18.5, RP11_405M12.2, and ADAM30 were significantly overexpressed in cancer tissues. These genes can be used as potential biomarkers of endometrial cancer and provide data support for precise immunotherapy in UCEC tumors.

## 2. Materials and Methods

### 2.1. Collection of Expression Profile and Clinical Data

Initially, the data on the expression level of UCEC patients as well as their clinical follow-up data were acquired from the TCGA database (https://portal.gdc.cancer.gov/). The following procedures are utilized to process the RNA-Seq data obtained from TCGA-UCEC: (1) samples that lacked clinical follow-up data were removed; (2) samples whose survival time was unknown, <30 days, and lacked survival status were removed; (3) the probes were turned into Gene Symbol; (4) if one probe corresponds to multiple genes, it was eliminated; (5) the median expression level is used for the Gene Symbol that contains multi-probes. After pretreatment, there are 542 tumor samples in the TCGA-UCEC data, and the clinical statistical information of samples is depicted in Table 1.

### 2.2. Consistent Clustering of Gene Expression Profiles Linked to Tumor RNA m5C

5-methylcytosine (m5C) is one of the important methylation modifications in RNA, and it is also a research hotspot in recent years. With the advent of methylation sequencing technologies, a substantial number of m5C methylation modifications in both coding RNA and non-coding RNA have been identified. The m5C methylation modification of RNA is regulated by m5C methyltransferase, demethylase, and m5C methylation binding protein. M5C methylation regulates the stability, transport, translation, and stress of RNA and participates in the process of tumor occurrence and development, invasion and metastasis, tumor drug resistance, and so on. For unsupervised clustering, the ConsensuClusterPlus package in R employed the Pam technique premised on Euclidean and ward linkage, which was performed 1000 times to guarantee the stability of categorization.

### 2.3. Differentially Expressed Genes between Tumor RNAm5C Subtypes (RNAm5C_DEGs)

Tumor samples were separated into two groups premised on the expression of RNAm5C-related genes and the findings of consistent clustering: RNAm5C-1 and RNAm5C-2. Utilizing the R software package limma, the DEGs across RNAm5C subtypes in TCGA-UCEC tumor samples were examined. Adjusted *p* < 0.05 and | log2 (Fold Change) | >1 served as the criteria for DEG screening. Furthermore, we employed the annotation file (∗.GTF) of the genome in the Ensemble to obtain the annotation in the DEGs.

### 2.4. Dimensionality Reduction of Gene Characteristics and Establishment of RNA Methylation Score (RS) Model

In this study, an RNA methylation score (RS) model of the tumor was constructed based on RNAm5C subtype-associated DEGs. First, a univariate cox technique was applied to minimize the size of the RNAm5C subtype-associated DEG set to remove noise or redundant genes. Following it, principal components analysis (PCA) was utilized to further minimize the dimension of variables and the number of genes within the risk model. Lastly, following PCA dimensionality reduction, the weight values of the first and second dimensions were utilized to generate the tumor RNA methylation score (RS) model, and the equation for its derivation is as follows:

(1) $$\begin{array}{c} \text{RS}=\sum \text{P}\text{C}1\left(\text{i}\right)+\sum \text{P}\text{C}2\left(\text{i}\right). \end{array}$$

### 2.5. Gene Set Enrichment Analysis (GSEA)

GSEA is a technique that was first described in a publication titled *Gene set enrichment analysis.* It is a technique for enrichment analysis that is premised on gene sets. When analyzing gene expression data, initially, we established the objectives of the study, which is conducted by selecting one or more functional gene sets from MSigDB for further investigation (gene matrix transposition file format ∗.gmt). Specifically, the association between the data on gene expression and the phenotype was used to determine the ranking (it may alternatively be viewed as the difference in the expression). Lastly, following the completion of the phenotypic correlation ranking, we examined each gene set to determine if its genes were enriched in the upper or lower portion of the gene list so that we can evaluate the impact that the coordinated variations in gene expression within this gene set had on the phenotypic variations.

### 2.6. Isolation of RNA and RT-PCR Analysis

At the Affiliated Hospital of Xi'an Jiaotong University, 16 pairs of human endometrial carcinoma samples along with the corresponding normal endometrial samples were obtained from different patients. The Ethics Committee of the Affiliated Hospital of Xi'an Jiaotong University granted its approval for the research project after obtaining permission from all of the patients who gave their informed consent. The TRIzol reagent (Invitrogen, Carlsbad, CA, USA) was utilized to isolate RNA from the tissues. Utilizing the QuantiTect Reverse Transcription Kit (Qiagen, Valencia, CA, USA), RNA was converted into cDNA by reverse transcription. SYBR Green (Takara, Otsu, Shiga, Japan) was employed for the quantification of the real-time PCR analyses and the values were subjected to normalization to the levels of GAPDH.

### 2.7. Analysis of Statistics and Hypothesis Confirmation

The statistical analysis technique in R 3.6 was utilized for all statistical comparisons in this research and for testing the significant differences across distinct groups. Survival curves were generated using the Kaplan-Meier method. The Wilcoxon test was used to compare the differences between two groups of samples, and the Kruskal-Wallis was used to compare the differences between multiple groups of samples, where ns means *p* > 0.05, ∗ means *p* < = 0.05, ∗∗ means *p* < = 0.01, ∗∗∗ means *p* < = 0.001, and ∗∗∗∗ means *p* < = 0.0001. Where *p* < 0.05 was considered significant difference with statistical significance.

## 3. Results

### 3.1. Molecular Features of UCEC Genes Involved in RNA Methylation (RNAm5C)

The analysis flow chart illustrates the general concept of analysis that was used in this investigation (Figure 1). Premised on the data set provided by TCGA-UCEC, we identified the mutations of 17 genes linked to RNA methylation (writers: TRDMT1, DNMT3B, DNMT3A, DNMT1, NSUN7, NSUN6, NSUN5, NSUN4, NSUN3, NSUN2, and NOP2; erasers; ALKBH1, TET3, TET2, and TET1; readers: YBX1 and ALYREF) (Figure 2(a)). It can be found that in the TCGA-UCEC data set, 17 RNA methylation-related genes have different degrees of mutations, among which TET1 (33%), TET3 (27%), TET2 (26%), DNMT1 (23%), and DNMT3B (23%) have higher mutations. After that, the copy number variation (CNV) of 17 genes linked to RNA methylation was analyzed and recorded (Figure 2(b)). In the TCGA-UCEC data set, it was discovered that there is a certain frequency of CNV, where the CNV of the TET1 gene is much more prevalent in contrast with other variations, accounting for over 30% of the total, and is primarily gain CNV.

At the transcriptomic level, comparisons were made to probe into the differences between normal and malignant tissues in the expression levels of 17 genes associated with RNA methylation (Figure 2(c)). The findings illustrated that a vast majority of genes have substantial variations in expression, in which NOP2, TET3, DNMT3B, DNMT3A, DNMT1, ALYREF are considerably up-modulated in tumor tissues, whereas NSUN3, NSUN6, TRDMT1, TET2, and ALKBH1 are remarkably down-modulated in tumor samples. At the protein modulation level, the network diagram of protein level interaction is drawn premised on the String database (https://www.string-db.org/) (Figure 2(d)). It has been discovered that genes interact with one another.

The prognostic value of 17 RNA methylation-related genes was further evaluated with the aid of the TCGA-UCEC data set. It can be found that most of the molecules have the value of prognostic risk factors with relatively significant significance (Figure 3).

### 3.2. Relationship of RNAm5C-Associated Genes with Immune Cell Infiltration (ICI) in UCEC

We employed CIBERSORT to assess the infiltration status of 22 distinct immune cells in the TCGA-UCEC data set to examine the association of RNAm5C-related gene expression with the tumor immune microenvironment (T.cells.CD4.naive, T.cells.CD8, Plasma.cells, B.cells.memory, B.cells.naive, T.cells.CD4.memory.resting, T.cells.CD4.memory.activated, T.cells.follicular.helper, T.cells.regulatory.Tregs, T.cells.gamma.delta, NK.cells.resting, NK.cells.activated, Monocytes, Macrophages.M0, Macrophages.M1, Macrophages.M2, Neutrophils Eosinophils, Mast.cells.activated, Mast.cells.resting, Dendritic.cells.activated, and Dendritic.cells.resting) (Table S1). Firstly, by analyzing the co-expression of RNAm5C-associated genes in the TCGA-UCEC data set (Figure 4(a)), it can be found that most genes show a significant positive correlation. Subsequently, the analysis of the link between the expression levels of 17 RNAm5C genes and the infiltration levels of 22 different types of immune cells (Figure 4(b)) showed that there were considerable variations across various genes and the infiltration levels of immune cells, where the SUN7 gene was substantially linked to the infiltration of a vast majority of immune cells. Utilizing the optimal density gradient approach, the samples in the TCGA-UCEC set were separated into two groups for the NSUN7 gene. The findings of the survival curves revealed a significant variation across the two groups. Patients in the NSUN7 low-expression group had a considerably longer overall survival (OS) in contrast with the high-expression group (Figure 4(c)). Similar trends can be seen in the survival analysis of progression-free survival, although the result was not significant (PFS) (Figure 4(d)).

The low- and high-expression profiles of the NSUN7 gene served as the basis for the GSEA that was performed. As depicted in Figure 4(e), the predominantly enriched pathways for the samples within the high-expression group were, respectively, SPLICEOSOME and UBIQUITIN MEDIATED PROTEOLYSIS. In the low-expression group, the predominantly enriched pathways were OLFACTORY TRANSDUCTION. Further, the effect of clinical features (Age, Grade, and Mutation.subtype) in the TCGA-UCEC data set on the expression of the NSUN7 gene was observed. As depicted in Figure 4(f), it was found that NSUN7 gene expression in the high-age group (age>65) has a certain upward trend, but no remarkable variation was identified in the expression of the NSUN7 gene in distinct tumor grade groups (Figure 4(g), Grade). In the grouping of different mutant subtypes, the expression level of the NSUN7 gene in cluster 3 was considerably elevated in contrast with that in cluster 1 (Figure 4(h)).

## 4. Detection and Functional Enrichment Analysis of RNAm5C Subtypes in UCEC

Consistent clustering was performed based on the expression patterns of 17 RNAm5C-associated genes for each sample of the TCGA-UCEC data set, and eventually, two distinct RNAm5C subtypes with substantial variations in survival status were found. Among the two primary RNAm5C subtypes, RNAm5C-2 led to a much more favorable prognosis in contrast with RNAm5C-1, with a median survival duration of over 6000 days. As illustrated in Figure 5, RNAm5C-2 is linked to a grim prognosis, with a median survival period of 3112 days.

To additionally examine the association of tumor RNAm5C subtypes with tumor immune cells, the PCA technique was utilized to display the RNAm5C-related expression pattern. In the space of the first and second dimensions, it was discovered that the samples had superior aggregation forms (Figure 6(a)), and the OS time between the three groups was significantly different (Figure 6(b)). It demonstrates that the RNAm5C subtype-related categorization approach is accurate and reliable.

Next, the variations in immune cell infiltration among the RNAm5C subtypes were compared (Figure 6(c)). The findings illustrated that regulatory T cells, CD8 positive T cells (T cellCD8), and plasma cells were significantly highly infiltrated in RNAm5C-2 subtypes. Moreover, the cells with significant high-level infiltration in the RNAm5C-1 subtype included M1 macrophages (Macrophages M1), M2 macrophages (Macrophages M2), and dendritic cells activated (Dendritic cells activated).

Further sequencing of genes was done as per the RNAm5C subtype, and the results of the sequencing were subjected to GSEA (Figure 6(d)). The pathways that had higher enrichment scores in RNAm5C-1 and RNAm5C-2 subtypes were RUNX1 REGULATES ESTROGEN RECEPTOR MEDIATED TRANSCRIPTION, TNFR1-INDUCED PROAPOPTOTIC SIGNALING, and HDMS DEMETHYLATE HISTONES, respectively. Pathways having higher enrichment scores in RNAm5C-3 subtypes include SENSORY PERCEPTION OF SALTY TASTE and IONOTROPIC ACTIVITY OF KAINATE RECEPTORS.

### 4.1. Immune-Associated Factor Expression across Tumor RNAm5C Subtypes

Signaling factors associated with the immune have a significant impact on the development of the tumor immune microenvironment, and it is important to conduct additional research on the link that exists between RNAm5C subtypes and immune signaling molecules present in tumors. Firstly, utilizing a heat map of genes linked to RNAm5C, we examined how each gene contributed to the categorization of RNAm5C phenotypes (Figure 7(a)). It has been established that the genes DNMT3A, DNMT1, DNMT3B, and YBX1 perform an integral function in the categorization process. Furthermore, by investigating the variations in the expression level of several immune-associated factors across the RNAm5C subtypes (Figure 7(b)), we discovered that there are substantial variations in a majority of categories, where Type II IFN Response, Pan-F-TBRS, EMT2, Immune checkpoint, Co-inhibition APC, MHC-II HLA, and Co-inhibition T cell exhibited an elevated level of the activation signal in RNAm5C-1 subtype. Through additional investigation of the variations in immune-associated factor expression that exist across phenotypes (Figure 7(c)), it can be found that most immune signal factors have significant differential expression.

The limma package of the R program was used to undertake an analysis of the gene expression patterns that differed among RNAm5C subtypes in TCGA-UCEC tumors to elucidate the possible biological properties of various RNAm5C states. Premised on adjusted *p* < 0.05 and | log2(Fold Change) | >1, which were applied as the screening cutoff values of DEGs, we discovered 711 DEGs (Table S2), where 590 genes were substantially up-modulated in the RNAm5C-2 subtype and 121 genes were substantially up-modulated in the RNAm5C-1 subtype, as displayed in Figure 7(d). Subsequently, the highly expressed genes identified from the various RNAm5C subtypes were examined for GO enrichment analysis, and a bubble diagram was utilized to depict the top ten enriched pathways in each of the three functional classes (BP, MF, and CC), as depicted in Figures 7(e)and 7(f). From the figure, it is apparent that the majority of the enriched pathways are linked to various kinds of biological pathways such as endopeptidase activity, proteolysis, mRNA splicing, and immunoglobulin regulation.

Univariate analysis was performed on 711 tumor RNAm5C subtype-related differentially expressed genes (DEGs), and further screened the prognostic DEGs. *p*.adjust <0.1 was set as the prognostic threshold. Finally, 34 prognostic DEGs were identified (Figure 8).

The 34 DEGs related to RNAm5C subtypes of tumors were obtained, and the expression profiles of DEGs were unsupervised clustered using the ConsensuClusterPlus tool in R. Furthermore, the TCGA-UCEC tumor samples were classified into five distinct gene subtypes (DEG.cluster), and there were significant survival differences between different gene subtypes, as shown in Figure 9.

### 4.2. Establishment of an RNA Methylation Score (RS) and Determination of Differential Gene Subtypes in Tumors

The PCA technique was utilized to narrow the dimensionality of the expression profile of differential genes premised on the DEGs across the RNAm5C subtypes. Lastly, the RNA methylation score (RS) was calculated by summing up the weights assigned to each sample in both the first and second dimensions. After that, the Survminer program in R was employed to compute the optimum density gradient cutoff value of tumor RNA methylation score (RS) associated with survival, where a score value of -0.8 was chosen to serve as the critical point in the analysis. In TCGA-UCEC, the tumor samples were separated into two groups, depending on their RS scores, and there was a remarkable variation in survival across the two groups, as shown in Figure 10.

Following that, the molecular properties of various gene subtypes were examined for the purpose of understanding the impact of tumor RNAm5C subtypes on genome-wide expression profiles. As depicted in Figure 11(a), the heat map illustrates how DEGs contribute to the grouping of differential gene subtypes.  Figure 11(b) illustrates substantial variations in the rates of survival across the various gene subtypes. When examining immune-related signal indicators, there are considerable differences in the expression of a majority of immune-associated factors across the various gene subtypes, as depicted in Figure 11(c).

Further, according to the analysis of the differences in RS among tumor mutation subtypes, RNAm5C subtypes, and different gene subtypes, as shown in Figures 11(d)–11(f), we can find that there are significant differences in RS among these groups. These findings might offer fresh perspectives on how to probe into the mechanisms behind tumor RNAm5C status and gene mutation in immune checkpoints.

## 5. Features of RNA Methylation Score (RS) in the Validation Data Set

The data sets GSE19041 and GSE17025 from the GEO database were chosen for analysis to additionally examine the reliability of RNA methylation score (RS) premised on differential gene establishment to predict the OS of patients with UCEC tumors. Firstly, the RS was computed for the data sets GSE19041 and GSE17025 based on the differential genes that had been screened in the preliminary step, and the Survminer program in R was utilized to perform the calculations necessary to determine the optimum density gradient cutoff value of tumor RS linked to survival. The tumor samples from the two different data sets were categorized into two groups as per their RS scores: low- and high-score groups (Figure 12(a)). As depicted in Figure 12(b), there were considerable variations in the rates of survival across the two groups with low and high scores, respectively. Further, the heat map illustrates the association that exists between clinical parameters and RS in the two GEO data sets. As may be seen in Figures 12(c) and 12(d), RS has a certain correlation with a variety of other clinical characteristics. Then, the differences in RS across different clinical features (Age, Grade, and Stage) groups were compared in GSE17025. The findings illustrated a substantial elevation in the risk score in the high-age group (age>65) (Figure 12(e)), the risk score in tumor grade Grade3 was considerably elevated as opposed to that in Grade1 (Figure 12(f)), and the risk score in tumor grade Stage IB was considerably elevated in contrast with that in Stage IA (Figure 12(f)).

### 5.1. Assessment of the Prognostic Significance of the Tumor RNA Methylation Score (RS) in Immunotherapy Efficacy

We evaluated the predictive performance of tumor RNA methylation score (RS) in determining the effectiveness of immunotherapy for patients. This research employed the IPS score of TCGA-UCEC samples included in the TCIA database as well as the IMvigor210 data set (http://researchpub.gene.com/IMvigor210CoreBiologies) and GSE18728 data set of immunotherapy queue for related assessment and analysis. The immunophenoscore (IPS) is a variable that may be used to measure the tumor's immunogenicity and anticipate how different kinds of cancers would respond to immunotherapy. As depicted in Figures 12(a)–(d), the 4 kinds of IPS scores (ips_ctla4_neg_pd1_neg, ips_ctla4_pos_pd1_neg, ips_ctla4_neg_pd1_pos, and ips_ctla4_pos_pd1_pos) in the high-RNA methylation score (High_RS) group were significantly elevated in contrast with those in the low-RNA methylation score (Low_RS) group (Figures 13(b)–(d)) except Figure 13(a), indicating that individuals with a high-RNA methylation score had a high likelihood of benefiting from immunotherapy as compared to those with a lower score. Patients who participated in the IMvigor210 clinical trial and were treated with anti-PD-L1 immunotherapy were assigned either a low- or a high-risk score (Figure 13(e)). It is important to point out that patients who were classified as having a high-RNA methylation rating (High RS) survived remarkably longer in contrast with those classified as having a low-RNA methylation rating (Low RS) (Figures 13(f)–13(h)). When compared with the low-RNA methylation evaluation group, the objective response rate of anti-PD-L1 therapy in the high-RNA methylation evaluation group was remarkably higher. In the IMvigor210 cohort, a greater level of RNA methylation is associated with an objective response to anti-PD-L1 therapy.

### 5.2. Identification of Biomarkers in Tumor RNA Methylation Risk Score (RS) Subtypes

Finding high-quality biological markers is crucial for further simplifying the accurate evaluation of tumor RNA methylation risk score subtypes in clinical practice. Hence, for the 34 DEGs between RNAm5C subtypes (RNAm5C_DEGs) with prognostic significance previously screened, a binary decision tree was established using the caret package and cross-validated (*k* =5), and the accuracy of classification was evaluated by specificity, sensitivity, and likelihood ratio (LR). The results show that MAGO3P is located at the root of the binary tree and has important decision-making abilities, as shown in Figure 14(a). Finally, eight genes were retained in the binary decision tree, namely, MAGOH3P, RP11_606P2.1, TRBJ2_3, CCT7P1, YTHDF1P1, RP11_323D18.5, RP11_405M12.2, and ADAM30. We further used PCR to validate the expression patterns of these genes in cancer tissues and adjacent tissues. The results showed that the six genes MAGOH3P, TRBJ2_3, YTHDF1P1, RP11_323D18.5, RP11_405M12.2, and ADAM30 were significantly overexpressed in cancer tissues. These genes can be used as potential biomarkers of endometrial cancer (Figures 14(b)–14(i)).

## 6. Discussion

The essence of tumorigenesis and development is the abnormal proliferation of cells, and this phenomenon is the result of abnormal cell proliferation caused by abnormal gene expression in cells. Studies done in the past have demonstrated that m5C modulatory factors exhibit a strong link to the growth and development of cells. Earlier research reports [22, 23] have also illustrated that the m5C regulator NSUN2 serves as the downstream target gene of oncogene MYC. MYC up-regulation facilitated the progression of the cell cycle as well as the up-regulation of NSUN2, and the highest expression was observed in the S phase. There is a substantial correlation between the NSUN2 expression and the clinical stage, progesterone receptor, estrogen receptor, pathological differentiation, tumor type, and Ki-67 expression profiles in breast cancer [23]. NSUNI has been recognized as a potential prognostic indicator in non-small cell lung cancer [24]. These results indicate that m5C regulatory factors may perform an integral function in tumors in different ways and may influence the prognosis of tumor patients by regulating the biological behavior of tumor cells. However, it is not clear how these regulatory factors work.

Therefore, we first observed the mutations of 17 RNA methylation-related genes (writers: TRDMT1, DNMT3B, DNMT3A, DNMT1, NSUN7, NSUN6, NSUN5, NSUN4, NSUN3, NSUN2, and NOP2; erasers: ALKBH1, TET3, TET2, and TET1; readers: YBX1 and ALYREF) in UCEC. The results showed that TET1 (33%), TET3 (27%), TET2 (26%), DNMT1 (23%), and DNMT3b (23%) had higher mutations. The study found that TET has mutations in a variety of tumors, and the highest mutation rate in this study is TET1, which has repeated mutations in a variety of cancers and is more common in skin cancer, lung cancer, gastrointestinal cancer, and urogenital cancer. Additionally, its mutation is positively linked to the efficacy of immune checkpoint inhibitors (ICIs) [25]. There is a possibility that genes linked to m5C might function in this manner. Subsequently, we explored gene CNV, of which the CNV of the TET1 gene is more prominent, accounting for over 30% (mainly gain copy number variation). However, whether this acquired CNV promotes the progress of UCEC needs further confirmation. Previous studies have disputed the role of TET1 in tumors. Studies have shown that TET1 inhibits colon cancer proliferation by impairing the *β*-catenin signaling pathway [26]. However, in hepatocellular carcinoma, TET1 up-regulation promotes the growth of cancer cells through the abnormal enhancer hydroxymethylation of HMGA2 [27], and in lung cancer, it also acts as a cancer-promoting gene to inhibit the aging of lung cancer cells by inhibiting the function of p53 [28]. This shows that the role of these genes in tumors is contradictory, which may also explain our results that some genes are highly expressed in tumors, but some are low expressed. However, after evaluating the prognostic value of these genes, it was found that most of the molecules have significant prognostic risk values. Almost all patients exhibiting a high expression of related genes have an unfavorable prognosis, indicating that they may all have cancer-promoting effects, but how they function needs further research.

In addition to the role of tumor cells themselves, the significance of the tumor microenvironment (TME) in the onset and progression of cancers has been demonstrated by an increasing number of research reports. Therefore, after conducting thorough research into the connection between the expression of associated genes and TME, we discovered that there was a significant variation between different genes and the infiltration levels of immune cells. The most prominent gene is the NSUN7 gene, which has a substantial link to the infiltration levels of most immune cells. In previous studies, it has been found that NSUN7 is a gene constituting the prognosis model of diverse tumors, such as prostate and lung cancers [29, 30], and is closely related to the TME. In the current research project, UCEC patients were categorized into two groups, the high- and the low-expression groups, premised on the level of the NSUN7 gene expression. The findings demonstrated that there was a remarkable difference in the survival curves between both groups. The OS rate of patients in the group with low expression was higher in contrast with those in the group with high expression. Similar trends can be seen in the survival analysis of PFS. It shows that even NSUN7 itself is a good prognostic gene of UCEC, and the previous result analysis shows that its mutation rate in UCEC is not high, indicating that the expression level of NSUN7 itself serves as a pathway in the tumor and its microenvironment. In addition, the low- and high-expression states of the NSUN7 gene were utilized as the basis for GSEA. It was found that in the high-expression state, the predominantly enriched pathways of samples were, respectively, SPLICEOSOME and UBIQUITIN MEDIATED PROTEOLYSIS, while in the low-expression state, the predominantly enriched pathways of samples were, respectively, OLFACTORY TRANSDUCTION. It shows that it participates in different pathways in tumorigenesis and development through abnormal expression, thus affecting the prognosis of tumors. Interestingly, it can be found that the expression of the NSUN7 gene has a certain up-regulation trend in the high-age group, although no remarkable variation was found in the expression of the NSUN7 gene in distinct tumor grade groups, and the high incidence age of UCEC was present in postmenopausal women. Whether this feature of NSUN7 is the starting mechanism of UCEC in postmenopausal women needs further exploration.

To better explore the function of RNAm5C-related genes in UCEC, we conducted consistent clustering according to the expression profile and finally discovered 3 distinct RNAm5C subtypes with considerable survival differences: RNAm5C-1, RNAm5C-2, and RNAm5C-3. The prognoses for patients belonging to each of these three subtypes are remarkably distinct from one another, with RNAm5C-2 leading to a prognosis that is remarkably superior to that of RNAm5C-1. We conducted further research on the link that exists between subtypes and immune cell infiltration to assess the factors that may contribute to the variation in prognosis. Multiple research reports illustrate that the TME includes immune cells (mast cells, dendritic cells, polymorphonuclear cells, macrophages, natural killer (NK), and T and B lymphocytes) and stromal cells, which perform a fundamental function in immunotherapeutic response, tumor progression, and immune evasion [31]. The results showed that regulatory T cells, CD8 + T cells, and plasma cells experienced substantial infiltration levels in the RNAm5C-2 subtype. In the RNAm5C-1 subtype, the cells with significant high-level infiltration comprise M1 macrophages, M2 macrophages, and activated dendritic cells. This could help explain, at least in part, why the prognosis for each of the three subtypes is significantly different. Research has illustrated that cd8+T cell infiltration is linked to a favorable prognosis [32], while the infiltration of M2 macrophage often predicts an unfavorable prognosis [33]. In addition, there are significant differences in the expression of immune-related factors in each subtype. Among them, the signal pathways such as MHC-II HLA, Type II IFN Response, Pan-F-TBRS, EMT2, Co-inhibition APC, Co-inhibition T cell, and Immune checkpoint have a high level of activation signals in RNAm5C-1 subtype. The activation of these signal pathways promotes tumor progression and inhibits the function of immune cells, which further explains why the prognosis of the RNAm5C-1 subtype is poor. In addition, the enrichment results of pathways in the three subtypes are different: The pathways with higher enrichment scores in RNAm5C-1 and RNAm5C-2 subtypes are RUNX1 REGULATES ESTROGEN RECEPTOR MEDIATED TRANSCRIPTION, TNFR1-INDUCED PROAPOPTOTIC SIGNALING, and HDMS DEMETHYLATE HISTONES. Pathways with higher enrichment scores in RNAm5C-3 subtypes include SENSORY PERCEPTION OF SALTY TASTE and IONOTROPIC ACTIVITY OF KAINATE RECEPTORS.

To further strengthen the clinical application value of RNAm5C-related genes, the gene differential expression between subtypes was analyzed, and the high-expression genes in different RNAm5C subtypes were analyzed for GO function enrichment. As per the findings, the majority of the enriched pathways were associated with biological pathways such as immunoglobulin modulation, endopeptidase activity, proteolysis, and mRNA splicing. Through univariate analysis of the differentially expressed genes (DEGs) related to the RNAm5C subtype, 34 differentially expressed genes with prognostic significance were finally identified. Based on these differential genes, the expression profile of differential genes was analyzed by dimensionality reduction, and the RNA methylation score (RS) was categorized into two groups: high- and low-RS score groups. In terms of prognosis differences, patients in the high-RNA methylation score group exhibited considerably longer survival time in contrast with those in the low-RNA methylation score group, and the objective response rate to anti-PD-L1 therapy in the high-RNA methylation score group was elevated in contrast with that in the low-RNA methylation score group, which provided a basis for clinical immunotherapy application and efficacy prediction. Finally, eight genes, MAGOH3P, RP11_606P2.1, TRBJ2_3, CCT7P1, YTHDF1P1, RP11_323D18.5, RP11_405M12.2, and ADAM30, remained in the binary decision tree. The findings of our PCR experiment provided additional evidence that the expression patterns of these genes are present in cancer cells as well as nearby tissues. The results showed that the six genes MAGOH3P, TRBJ2_3, YTHDF1P1, RP11_323D18.5, RP11_405M12.2, and ADAM30 were significantly overexpressed in cancer tissues. These genes can be used as potential biomarkers of endometrial cancer. The current research on these genes is limited, among which TRBJ2_3 is a kind of T cell TCR, which can regulate T cell function to a certain extent [34]; RP11_323D18.5 and RP11_405M12.2 were long-chain non-coding RNA related to m6A modification.

Nevertheless, there are still some limitations to this research. First of all, we only applied UCEC samples in the TCGA database and could not carry out strict inter-group condition control, which may lead to deviation in the study of m5C RNA methylation modulators and clinical-pathological characteristics, and lack of verification of real clinical data. Secondly, notwithstanding the exploration of the link between differential genes and immune cells, the clinicopathological characteristics were not associated with the infiltration status of immune cells, which were extremely related to the occurrence, development, and prognosis of tumors. In addition, PCR was only employed to confirm the expression of the finally screened prognosis-related genes, and the protein level and specific biological function were not verified. Third, the role of the relevant signal pathways screened in UCEC is not clear. Fourth, the small sample size in the current research necessitates more research to reinforce and confirm the stability of the risk model. Further research and trials in the field of molecular biology are warranted.

## 7. Conclusions

In summary, the majority of m5C RNA methylation modulators experience an aberrant expression in UCEC. M5C regulator has prognostic value. These modulators influence the tumor immune microenvironment, which is directly linked to the onset and progression of UCEC. Therefore, the m5C RNA methylation modulator may become a prognostic marker of UCEC.

## Figures and Tables

**Figure 1:** Analysis flow chart.

**Figure 2:** Multi-omic features of 17 RNAm5C-associated genes in the TCGA-UCEC data set. (a) Waterfall diagram of gene mutation. (b) Bar graph of gene copy number variation. (c) Box diagram of gene expression difference between normal and tumor tissue. (d) Interaction network of genes at the protein level.

**Figure 3:** Survival curves of 17 RNAm5C-related genes in TCGA-UCEC data set.

**Figure 4:** The relationship between RNAm5C gene and the infiltration status of tumor immune cells in TCGA-UCEC data set. (a) Gene co-expression loop. (b) A heat map showing the association between 22 different types of immune cell infiltration and the corresponding genes. (c, d) Survival analysis of OS and PFS with high and low gene expression in TCGA-UCEC data set. (e) Gene set enrichment analysis under low and high gene expression. (f, g, h) Differences in the expression of NSUN7 gene in different clinical groups (Age, Grade, Mutation. subtype) in TCGA-UCEC data set.

**Figure 5:** Consistent clustering of gene expression profiles associated with tumor RNAm5C. (a, b, c, d) The findings from clustering based on the classification number *k* =2, *k* =3, *k* =4, *k* =5. (f, g, h, i) Survival curve based on the classification number *k* =2, *k* =3, *k* =4, *k* =5. (e) CDF curve showing consistent clustering distribution. (j) The distribution of the area under the CDF curve of consistent clustering.

**Figure 6:** Determination and functional enrichment analysis of RNAm5C subtypes within the TCGA-UCEC data set. (a) PCA analysis of RNAm5C gene set. (b) Survival curve between tumor RNAm5C subtypes. (c) The variation of 22 kinds of immune cell infiltration between tumor RNAm5C subtypes. (d) Analysis of pathway enrichment of gene sets with differential expression across RNAm5C subtypes.

**Figure 7:** Variations in the expression of immune-related factors across tumor RNAm5C subtypes. (a) Heat map of 17 RNAm5C gene expression profiles. (b) Variations in immune-associated factor sets across tumor RNAm5C subtypes. (c) Differential expression of immune-related factors among tumor RNAm5C subtypes. (d) Volcanic map of differential expression analysis between tumor RNAm5C subtypes. (e) Analysis of Go enrichment of downregulated gene sets across tumor RNAm5C subtypes. (f) Analysis of Go enrichment of up-regulated gene sets between tumor RNAm5C subtypes.

**Figure 8:** Univariate analysis of differentially expressed genes across tumor RNAm5C subtypes.

**Figure 9:** A consistent clustering of genes with differential expression across tumor RNAm5C subtypes. (a, b, c, d) The findings of clustering analysis based on the classification number *k* =2, *k* =3, *k* =4, *k* =5. (f, g, h, i) Survival curve when classification number *k* =2, *k* =3, *k* =4, *k* =5. (e) CDF curve distribution of consistent clustering. (j) The distribution of the area under the CDF curve of consistent clustering.

**Figure 10:** The optimum gradient classification of tumor RNA methylation (RS). (a) The statistical analysis of RS distribution density and the identification of the optimum threshold. (b) A survival curve between the high-RS group and the low-RS subgroup.

**Figure 11:** Identification and characteristic analysis of different gene subtypes. (a) Heat map of differential gene expression profile. (b) Survival curve among different gene subtypes. (c) Difference analysis of immune signal factors among different gene subtypes. (d, e, f) Differences in RNA methylation scores (RS) among RNAm5C subtypes (Sig. cluster), differential gene subtypes (DEG.cluster), and mutation subtypes (mutation. subtype). (g) A dynamic flow diagram depicting the grouping of tumor samples and the transition between states.

**Figure 12:** Tumor RNA methylation score-related characteristics in external data sets. (a) Identification of the best grouping threshold of the risk score in GSE119041 data. (b) The risk score-related survival curve in the GSE119041 data. (c, d) The relationship between risk score distribution and clinical diagnosis distribution in GSE119041 and GSE17025 data sets. (e, f, g) The variations of risk scores in distinct Grade, Age, and Stage groups of GSE119041 data set.

**Figure 13:** The function of the tumor RNA methylation score (RS) in the anticipation of whether or not immunotherapy would be beneficial. (a, b, c, d) The variations between low- and high-RS groups in terms of four different types of immunophenoscore (IPS) scores. (e) Variations in risk scores across various treatment response groups included in the IMvigor210 cohort. (f) The best density gradient method identifies the grouping threshold. (g) Variations in the proportion of various treatment response groups in the IMvigor210 cohort among patients with low- and high-risk scores. (h) Survival curve in the IMvigor210 queue among patients with low and high ICI scores.

**Figure 14:** Identification of biomarkers using binary decision tree. (a) Fork decision tree of candidate markers. (b–i) PCR tissue validation of candidate markers.

**Table 1:** Clinical information statistics of TCGA-UCEC data set.

	TCGA-UCEC
Survival	
OS	
Dead	92
Censored	450
Age	
Age>65	236
Age<=65	304
Age_UN	2
Histology	
Endometrioid endometrial adenocarcinoma	406
Mixed serous and endometrioid	22
Serous endometrial adenocarcinoma	114
Grade	
G1	98
G2	117
G3	313
High grade	11
Stage	
Stage_I	339
Stage_II	51
Stage_III	123
Stage_IV	29
Mutation.Subtype	
Cluster 4	73
Cluster 1	37
Cluster 3	30
Cluster 11	25
Others	377
Subtype	
Cluster 1	96
Cluster 2	104
Cluster 3	80
Cluster 4	90
Others	172

## Data Availability

The data used to support the findings of this study are available from the corresponding author on reasonable request.

## Supplementary Materials

Supplementary Materials Table S1. The infiltration status of 22 distinct immune cells in the TCGA-UCEC data set. Table S2.711 DEGs identified among RNAm5C subtypes.
